This article has been retracted.

# Study of Scraping with Copper Stone Based on Theory of Midnight-Noon Ebb-Flow in Angina Pectoris with Coronary Heart Disease of Qi Stagnation and Blood Stasis

**DOI:** 10.1155/2021/2677696

**Published:** 2021-09-18

**Authors:** Xianwen Tang, Jinguo Yang, Zhong Feng, Jingyu Piao, Quanhao Yan, Chao Gao

**Affiliations:** ^1^Department of Cardiology, Shenzhen Hospital of Beijing University of Chinese Medicine (Longgang), Shenzhen, Guangdong 518116, China; ^2^Guangdong Pharmaceutical University, Guangzhou, Guangdong, China

## Abstract

Angina pectoris (AP) with coronary heart disease (CHD) is one of the common cardiovascular diseases in clinical practice, which can be classified as “chest paralysis” in Chinese medicine according to its symptoms, and it is described in many ancient documents. Ancient Chinese medicine believes that the main pathogenesis of the disease is poor blood flow leading to paralysis of the heart and veins, so it is often treated by activating blood and removing blood stasis. In this study, 120 patients with AP of CHD of Qi stagnation and blood stasis type were randomly divided into the observation (*n* = 60) and the control group (*n* = 60). In the control group, basic care, conventional treatment, and unselected copper acupuncture scraping were used, while in the observation group, copper acupuncture scraping was performed at the right time of the heart meridian (11 : 00–13 : 00) on the basis of the control group, and all patients received the treatment for a total duration of 4 weeks. We collected data on the traditional Chinese medical (TCM) syndrome score, frequency and duration of angina attacks, nitroglycerin dosage, inflammatory factor levels, and hematological indices pretreatment and posttreatment in both groups. Patients' adverse effects during treatment were recorded, and the clinical efficacy and ECG efficacy in both groups were evaluated after 4 weeks. We used SPSS.20 statistical software to statistically analyze the above data, and the results showed that the clinical efficacy and ECG efficacy of the observation group were significantly higher than the control group posttreatment. After treatment, the TCM symptom score, angina attack frequency, attack duration and nitroglycerin dosage, serum interleukin-8 (IL-8), hypersensitive C-reactive protein (hs-CRP), and tumor necrosis factor-*α* (TNF-*α*) levels, whole blood viscosity (WBV), plasma viscosity (PV), fibrinogen (FIB), and hematocrit (Hct) were significantly lower in both groups compared with those posttreatment. And the observation group showed a greater decrease when compared with the control group. The results also showed that the overall incidence of adverse reactions was lower in both groups during the treatment period. The above results indicate that while ensuring high safety, the copper stone based on theory of midnight-noon ebb-flow can more effectively improve the symptoms and inflammatory response of the body and reduce the viscosity of the blood in AP with CHD of Qi stagnation and blood stasis, and it has better therapeutic effects.

## 1. Introduction

Angina pectoris (AP) with coronary heart disease (CHD) is a series of chest pain syndromes caused by atherosclerosis of the patient's coronary arteries, resulting in myocardial ischemia and hypoxia, with symptoms manifesting as recurrent episodes of crushing pain at the posterior sternal location, and is a common clinical cardiovascular disease [1, 2]. The incidence of CHD is quite high in the Chinese population, and modern medicine regarding the treatment of CHD is still based on multifaceted comprehensive treatment, which includes conservative medical drugs, PCI and CABG [3]. The recurrence rate of CHD with AP remains high despite the many approaches available, so it is urgent and necessary to actively search for new effective drugs and treatments.

CHD with AP belongs to the category of “thoracic obstruction” in traditional Chinese medicine (TCM), which has been described in many works, and TCM has a long history of efficacy in the prevention and treatment of this disease [4, 5]. The theory of midnight-noon ebb-flow originated from Huangdi's Classic on Medicine, which is guided by the idea of “nature-human integration” and believes that the strength of human Qi and blood corresponds to the natural circadian rhythm [6]. When copper acupuncture scraping therapy (Gua Sha) acts on human meridians, it can achieve the effects of unblocking the meridians, promoting blood circulation, eliminating blood stasis, detoxifying evil, tonifying Qi, and benefiting blood. Modern medicine believes that Gua Sha therapy has anti-inflammatory, antioxidant, immune enhancement, microcirculation improving, and neuromodulation stimulating effects on the human body [7, 8]. The Gua Sha therapy based on the theory of midnight-noon ebb-flow is in accordance with the relationship between the meridians of the human body and the twelve two-hour periods of the day, the selected meridians are scraped during specific times, and the combination of points, lines, and surfaces can effectively stimulate multiple areas at the same time.

We have been treating patients with AP of CHD for many years and have accumulated rich clinical experience by using TCM methods such as Gua Sha and foot baths. The patients with Qi stagnation and blood stasis (chronic stable AP) were selected as the subjects of this study and treated with scraping with copper stone base on the theory of midnight-noon ebb-flow and achieved good efficacy.

## 2. Data and Methods

### 2.1. Research Objectives

120 patients with AP of CHD admitted to Department of Cardiology, Shenzhen Hospital of Beijing University of Chinese Medicine (Longgang), from March 2018 to October 2019 were selected and randomly divided into observer and control groups, with 60 cases in each group. The comparison of baseline data of the two groups of patients, such as gender, age, course of disease, and comorbidities, is given in Table 1.

### 2.2. Inclusion Criteria

The inclusion criteria were as follows. Patients with a clear history of CHD. Patients who met the diagnostic criteria of Western medicine for chronic stable AP [9]: Chest pain is located in the upper middle part of the sternum or the precordial area, with a feeling of suffocation and obstruction, chest pain mostly occurring after exertion, emotional excitement, cold, and satiety, and lasts 3–5 min. Patients can relieve symptoms by taking nitroglycerin, and there are transient changes in the electrocardiogram. Patients aged from 45 to 80 years. TCM syndrome differentiation belonged to Qi stagnation and blood stasis type: the main symptoms are characterized by chest tightness and distension mostly triggered by emotional discomfort, frequent sighing, and distension in both sides of the abdomen, which can be somewhat relieved after belching or farting. The tongue and pulse are characterized by purple or dark red tongue and string pulse. Patients with informed consent and voluntary participation in the study.

### 2.3. Exclusion Criteria

The exclusion criteria were as follows. Patients with acute coronary syndrome, patients with combined malignancies, severe impairment of other vital organ functions, patients with hematological diseases and infectious diseases, patients who were intolerant to scrape therapy or had damaged local skin and have skin diseases, patients who were pregnant or breastfeeding and with poor treatment compliance, and neurological and mental disorders.

### 2.4. Treatment Methods

1. Control group: basic care of angina pectoris, conventional treatment, and unselected copper acupuncture scraping were used. The basic nursing care included instructing patients to pay attention to bed rest, avoid overexertion, keep warm, regulate diet, and prohibit smoking and alcohol. Routine treatment included vasodilatation, blood supply improvement, blood pressure and lipid lowering, anticoagulation, anti-inflammatory, and antioxidant treatment. The specific operation of copper acupuncture was as follows: assessing the patient's skin condition and determining the degree of pain tolerance, the patient took the sitting position and fully exposed the neck and back. After routine disinfection, Li's copper squash scraping board was used in conjunction with the scraping oil to operate, performing scraping with copper acupuncture: scraping Governor's meridian (Dazhui to Zhiyang acupoint) and bladder meridian (Xinshu to Geshu acupoint) first and then Ren channel (Danzhong to Zhongting acupoint) and pericardial meridian (Quze to Neiguan, Xi Men to Neiguan acupoint). The technique should be slow, the time should be short, and the strength should be small, based on patient tolerance. Scraping was performed 2 times/week for a 4-week course of treatment, with the duration of treatment variable and at the convenience of the patient. During the treatment period, one case was removed and detached.
2. Observer group: received the same basic care and conventional treatment as the control group. In conjunction with the theory of midnight-noon ebb-flow, we chose the right time of the heart meridian (11 : 00–13 : 00) and fixed the treatment for the patients at this time, and the scraping process, techniques, frequency, and duration of treatment were the same as the control group. During the treatment period, 4 cases were eliminated and shed.

### 2.5. Observed Indicators

1. The TCM symptoms scores were recorded pretreatment and posttreatment in both groups: the symptoms of chest pain, chest tightness, palpitations, and shortness of breath were rated as 0, 1, 2, and 3 according to none, mild, moderate, and severe, where none indicates no seizures of symptoms, mild indicates occasional seizures with mild symptoms, moderate indicates frequent seizures but mild symptoms, and severe frequent seizures with severe symptoms
2. The mean daily frequency of angina attacks, mean duration of each attack, and nitroglycerin dosage were recorded for 1 week pretreatment and posttreatment in both groups
3. Inflammatory factors and blood rheology indexes were measured and recorded pretreatment and posttreatment in both groups: 3–5 ml of fasting venous blood was drawn from patients, and we used the enzyme-linked immunosorbent assay to detect interleukin-8 (IL-8), hypersensitive C-reactive protein (hs-CRP), and tumor necrosis factor-*α* (TNF-*α*), and the relevant kits were purchased from Hangzhou Haoxin Biotechnology Co. Whole blood viscosity (WBV), plasma viscosity (PV), fibrinogen (FIB), and hematocrit (Hct) were determined using the LA-2a fully automated hematocrit analyzer.
4. The occurrence of adverse reactions during treatment in both groups was observed and counted: the adverse reactions included swelling, fatigue, subcutaneous bleeding, pain, nausea and vomiting, and chilling of the extremities.

### 2.6. Judgment of Efficacy [9]

After 4 weeks of treatment, we evaluated the clinical and ECG efficacies of the patients, as described in the following.

#### 2.6.1. Clinical Efficacy

The disappearance or almost disappearance of angina pectoris symptoms indicated that the treatment effect was significant, which was markedly effective. The obvious reduction of angina pectoris symptoms indicated that the treatment had a certain effect as valid. Angina pectoris symptoms were not improved as invalid.

#### 2.6.2. Efficacy of ECG

Markedly effective: the patient's ECG returned to normal or approximately normal at rest, and the double secondary gradient exercise test changed from positive to negative. Valid: patient's ST-segment decreased on ECG at rest or on the double 2-step exercise test, recovered more than 0.05 mV posttreatment but did not reach normal, in major led inverted T-segment becomes shallow by more than 50%, or T-wave changed from flat to upright. Invalid: the patient's ECG at rest or the double 2-step exercise test was essentially the same as before treatment or improved but did not meet the criteria for effectiveness.

Total efficiency rate = (markedly effective + valid) number of cases/total cases × 100%.

### 2.7. Statistical Methods

SPSS 20.0 software was used for data processing, and GraphPad prism 8 was used to make statistical graphs. Measurement data were expressed as mean ± standard deviation ($\bar{x}$±*s*), the independent sample *t*-test was used for comparison between groups, count data was expressed as (*n* (%)), and the chi-square (*χ*^2^) test was performed. *P* < 0.05 indicated that the difference was statistically significant.

## 3. Results

### 3.1. Comparison of Case Information between the Two Groups Pretreatment

Our statistical analysis of the general data of the two groups showed that there was no statistical difference between the two groups in terms of gender, age, disease duration, and comorbidities (*P* > 0.05, Table 1).

### 3.2. Comparison of Clinical Efficacy

Finally, 59 patients in the control group and 56 patients in the observation group completed the full course of treatment. The results of the efficacy analysis showed that the difference in total clinical efficiency between the two groups was statistically significant (*P* ＜ 0.05, Figure 1).

### 3.3. Comparison of ECG Efficacy

By comparing the difference in the total effective rate between the two groups, we found that the observation group was significantly higher than the control group (*P* ＜ 0.05, Figure 2).

### 3.4. Comparison of TCM Evidence Scores and AP Related for Pretreatment and Posttreatment

There was no statistical difference in the TCM symptom score, frequency and duration of angina attacks, and nitroglycerin dosage between the two groups pretreatment (*P* > 0.05). After each of the treatment, the TCM symptom scores, frequency and duration of angina attacks, and nitroglycerin dosage were significantly lower in both groups, with a greater decrease in the observer group (*P* < 0.05, Figure 3).

### 3.5. Comparison of Inflammatory Factor Concentrations for Pretreatment and Posttreatment

There was no statistical difference in serum IL-8, hs-CRP, and TNF-*α* concentrations between the two groups pretreatment (*P* > 0.05). After each of the treatment, the serum IL-8, hs-CRP, and TNF-*α* concentrations were significantly lower in both groups, with a greater decrease in the observer group (*P* < 0.05, Figure 4).

### 3.6. Comparison of Blood Flow Indexes for Pretreatment and Posttreatment

There was no statistical difference in WBV, PV, FIB, and Hct level between the two groups pretreatment (*P* > 0.05). After each of the treatment, the level of WBV, PV, FIB, and Hct was significantly lower in both groups, with a greater decrease in the observer group (*P* < 0.05, Figure 5).

### 3.7. Comparison of the Occurrence of Adverse Reactions

During the treatment period, 1 case of pain and 2 cases of swelling occurred in the control group, and the incidence of adverse reactions was 5.08% (3/59), while 1 case of pain and 1 case of swelling occurred in the observer group, and the incidence of adverse reactions was 3.57% (2/56), and the incidence of adverse reactions in the two groups was not statistically significant (*P* > 0.05, Figure 6).

## 4. Discussion

AP is one of the main types of CHD with irregular episodes and pain radiating to the shoulder and neck during attacks. Factors such as overwork, mood disorders, and climate change are potential triggers for the development of the disease, and if not treated in a timely manner, there is a high risk of developing acute myocardial infarction which may lead to a significant increase in the risk of death [10, 11]. Pharmacological treatment is a conventional therapy in Western medicine, which mainly focuses on 3 aspects: dilating diseased blood vessels, improving atherosclerosis, and lowering blood pressure, with the purpose of reducing myocardial oxygen consumption, delaying atherosclerotic lesions, improving myocardial blood supply, and thus relieving angina symptoms and reducing mortality [12]. AP of CHD is called “thoracic obstruction” in TCM theory, and the mechanism of the disease is paralysis of the heart arteries due to poor blood flow, so TCM doctors mostly use the method of activating blood and removing blood stasis for treatment. Gua Sha has the efficacy of promoting blood circulation, regulating Qi and draining the meridians, and is a characteristic TCM method to assist in the treatment of AP in CHD. With many years of experience in the field of TCM treatment, our institute is skilled in mastering and applying the skills of Gua Sha, which can ensure the smooth conduct of this study.

The location of thoracic obstruction is in the heart. A relevant description in the Zhu Bing Yuan Hou Lun reveals that the disease belongs to the evidence of deficiency of the root and the symptoms of the symptoms [13]. TCM emphasizes syndrome differentiation and treatment. The type of Qi stagnation and blood stasis selected for this study is one of the main types of thoracic obstruction. In ancient TCM, the heart is the master of the blood vessels and runs Qi and blood in the meridians to moisten the body; if the heart Qi sinks, it is difficult to move Qi and blood, fluid stagnation, Qi blockage, blood flow is not smooth accumulation of stasis, retention in the meridians, paralysis blocking chest yang, and inaccessibility of the heart chakra develops into thoracic obstruction [14–16]. The occurrence of Qi stagnation and blood stasis type of thoracic obstruction begins with the sinking of heart Qi. Based on the principle that the root cause of the disease needs to be found when treating the disease, this study selected the right time of the heart meridian (11 : 00–13 : 00) for Gua Sha treatment according to the theory of midnight-noon ebb-flow. The results showed that the clinical effective rate and ECG effective rate of the observation group were 89.29% and 92.86%, respectively, which were higher than those of the control group, indicating that scraping with copper stone under the guidance of the theory of midnight-noon ebb-flow had positive significance in improving the therapeutic effect. It should be noted that since the treatment needs a certain duration, the patients may have interrupted the trial for personal reasons. Therefore, before the study, the author explained the treatment process and requirements to the patients in detail to improve their compliance. After treatment, the TCM symptom scores, angina attack frequency, attack duration, and nitroglycerin dosage were lower in both groups than pretreatment, with the observer group being lower. It indicates that Gua Sha with copper stone can effectively relieve the symptoms of AP, and the therapeutic effect is better after combining with the theory of midnight-noon ebb-flow. Analyzing the reasons, the theory of midnight-noon ebb-flow believes that the blood Qi in different meridians should be full from time to time, and blood Qi should be decayed when it is out of date. Therefore, the heart meridian duty time is selected for treatment according to the concept of “adapt to the time and cure at the tim.” Through the technique of scraping with copper stone, we can activate the blood to remove blood stasis, regulate Qi, and broaden the chest, dredge the meridians and channels, so that Qi and blood can penetrate deep into the internal organs, thus achieving the purpose of improving the symptoms of angina pectoris [17, 18]. In addition, compared with the conventional Gua Sha tool, the Gua Sha tool used in this study is the Tiger Charm Copper Bian stone Scraping Board of Teacher Li Daozheng. Its unique brass texture enables it to achieve a better resonance frequency with the human body, so its heating effect, the effect of removing blood stasis, and the depth of energy penetration are greatly improved, so it can effectively act on the human body and enhance the therapeutic effect.

The inflammatory response is involved in the development of cardiovascular disease [19]. Inflammatory factors such as IL-8 and TNF-*α* are biopolymphatic, where IL-8 is not only associated with increased inflammatory cells but also induces smooth muscle cell proliferation, proliferating atheromatous plaques and increasing the risk of revascularization. TNF-*α* is an important mediator of the inflammatory response and has a promotional significance for coagulation. hs-CRP belongs to the acute temporal phase proteins and is a sensitive indicator of inflammation in the organism [20, 21]. The results of this study showed that the levels of IL-8, hs-CRP, and TNF-*α* were lower in the observer group than in the control group after treatment, suggesting that Gua Sha with copper stone based on the theory of midnight-noon ebb-flow may reduce the risk of cardiovascular events by reducing the inflammatory response. The reason for this analysis may be the direct stimulation of the skin by Gua Sha, which activates vascular and lymphatic circulation, improves blood perfusion, enhances intracellular metabolism, and promotes repair of damaged tissues [22]. Hemorheology indicators are serum markers that indicate cardiovascular events. The combined detection of WBV, PV, FIB, and Hct can reflect blood viscosity to a certain extent and is closely related to the pathological progress of atherosclerosis [23], [24]. In the present study, WBV, PV, FIB, and Hct were reduced in both groups posttreatment compared to pretreatment, with the observer group being lower than the control group, suggesting that Gua Sha with copper stone based on the theory of midnight-noon ebb-flow may alleviate angina symptoms by reducing blood viscosity. In addition, a detailed medical history should be obtained from the patient before scraping, and the physiological condition of the patient should be paid attention to at all times during scraping to avoid serious adverse reactions. In this study, the adverse reactions were mild in both groups and were effectively relieved after symptomatic care.

## 5. Conclusion

Combined with the contents of the text, we found that Gua Sha with copper stone based on the theory of midnight-noon ebb-flow for the treatment of AP with CHD of Qi stagnation and blood stasis could improve the efficacy and symptoms of angina pectoris, reduce the inflammatory response, lower the blood viscosity, and have high safety, and we concluded that the change of the treatment plan is worth to be promoted to clinical application.

## Figures and Tables

**Figure 1:** Comparison of clinical efficacy, compared with the total effective rate of the control group, ^*∗*^*P* < 0.05.

**Figure 2:** Comparison of ECG efficacy, compared with the total effective rate of the control group, ^*∗*^*P* < 0.05.

**Figure 3:** Comparison of TCM evidence scores and AP related for pretreatment and posttreatment. (a) Comparison of mean TCM symptom scores. (b) Comparison of mean AP attack frequency. (c) Comparison of mean seizure duration. (d) Comparison of mean nitroglycerin dosage. Compared with the same group pretreatment, ^^^*P* < 0.05. Compared with the control group posttreatment, ^*∗*^*P* < 0.05.

**Figure 4:** Comparison of inflammatory factor concentrations for pretreatment and posttreatment. (a) Comparison of mean IL-8 concentrations. (b) Comparison of mean hs-CRP concentrations. (c) Comparison of mean TNF-*α* concentrations. Compared with the same group pretreatment, ^^^*P* < 0.05. Compared with the control group posttreatment, ^*∗*^*P* < 0.05.

**Figure 5:** Comparison of blood flow indexes for pretreatment and posttreatment. (a) Comparison of mean WBV. (b) Comparison of mean PV. (c) Comparison of mean FIB level. (d) Comparison of mean Hct percentages. Compared with the same group pretreatment, ^^^*P* < 0.05. Compared with the control group posttreatment, ^*∗*^*P* < 0.05.

**Figure 6:** Comparison of the occurrence of adverse reactions.

**Table 1:** Comparison of general data of the AKI group and health group.

Data	Control group (*n* = 60)	Observer group (*n* = 60)	*P* value
Gender (case, %)			
Male	36 (60.00)	32 (53.33)	0.527
Female	24 (40.00)	27 (46.67)	

Basic diseases (case, %)			
Diabetes	12 (20.00)	11 (18.33)	0.817
Hypertension	19 (31.67)	20 (33.33)	0.948
Age, mean (SD), year	55.27 ± 9.55	56.15 ± 10.51	0.632
Disease duration, mean (SD), year	5.85 ± 2.38	6.07 ± 2.25	0.604

## Data Availability

The data used to support the findings of this study are available from all the authors upon request.
